# Application of Clustering-Based Analysis in MRI Brain Tissue Segmentation

**DOI:** 10.1155/2022/7401184

**Published:** 2022-08-03

**Authors:** Mingjiang Li, Jincheng Zhou, Dan Wang, Peng Peng, Yezhao Yu

**Affiliations:** ^1^School of Computer and Information, Qiannan Normal University for Nationalities, Duyun 558000, China; ^2^Key Laboratory of Complex Systems and Intelligent Optimization of Guizhou Province, Duyun 558000, China; ^3^School of Mathematics and Statistics, Qiannan Normal University for Nationalities, Duyun 558000, China; ^4^School of Artificial Intelligence and Computer Science, Jiangnan University, Wuxi 214122, China; ^5^School of Physics and Electronics, Qiannan Normal University for Nationalities, Duyun 558000, China

## Abstract

The segmentation of brain tissue by MRI not only contributes to the study of the function and anatomical structure of the brain, but it also offers a theoretical foundation for the diagnosis and treatment of brain illnesses. When discussing the anatomy of the brain in a clinical setting, the terms “white matter,” “gray matter,” and “cerebrospinal fluid” are the ones most frequently used (CSF). However, due to the fact that the human brain is highly complicated in its structure and that there are many different types of brain tissues, the human brain structure of each individual has its own set of distinctive qualities. Because of these several circumstances, the process of segmenting brain tissue will be challenging. In this article, several different clustering algorithms will be discussed, and their performance and effects will be compared to one another. The goal of this comparison is to determine which algorithm is most suited for segmenting MRI brain tissue. Based on the clustering method, the primary emphasis of this research is placed on the segmentation approach that is appropriate for medical brain imaging. The qualitative and quantitative findings of the experiment reveal that the FCM algorithm has more steady performance and better universality, but it is necessary to include the additional auxiliary conditions in order to achieve more ideal outcomes.

## 1. Introduction

MRI brain tissue segmentation, as we are all aware, not only contributes to the study of the function and anatomical structure of the brain, but it also offers a theoretical foundation for the diagnosis and treatment of brain illnesses [1]. Therefore, the achievement of precise tissue segmentation using MRI carries with it extremely significant implications for clinical diagnosis and treatment [2]. Within the context of medical practice, the segmentation of brain tissue primarily relates to the white matter (WM), gray matter (GM), and cerebrospinal fluid (CSF). However, due to the fact that the human brain is highly complicated in its structure and that there are many different types of brain tissues, the human brain structure of each individual has its own set of distinctive traits [3]. Because of these several circumstances, the process of segmenting brain tissue will be challenging. As a result, the development of an outstanding segmentation algorithm that is appropriate for every MRI brain tissue is a topic that presents a significant amount of difficulty. While doing so, it also encourages researchers to work on developing algorithms for segmenting brain tissue, which has become a primary focus of research in recent years [4, 5]. In clinical practice, it is frequently required to present a three-dimensional model of the structure of brain tissue in order to offer a foundation for the diagnosis and treatment of a patient. When brain surgery, for instance, is required, the procedure can be planned and simulated in accordance with the three-dimensional anatomy of the brain. This makes it easy for focus to quickly and accurately select the surgical area. In addition, the goal of visualizing brain tissue is to finish the job of segmenting it, which is the concept of visualization. Therefore, the segmentation of brain tissue has significant practical significance in the context of medical diagnostics [6–8].

Research on brain images is extremely vital to the progression of humankind; among the many key research paths being pursued, one that has garnered a lot of attention is the segmentation of brain tissue. It has, from the beginning, been understood to be a challenging issue to resolve on account of the intricate make-up of the brain as well as other aspects. After years of research, various segmentation algorithms are being applied to medical photos all around the world, including the United States. In general, medical image segmentation algorithms can be broken down into the following categories: threshold-based segmentation [9–11], edge detection-based segmentation [12–14], fuzzy-clustering-based segmentation [15], level-set-based segmentation [16, 17], and region-growth-based segmentation [18]. Each of these categories is named after a different method of segmentation.

A method known as threshold-based segmentation is a technique that can divide an image into its component parts. Its segmentation principle splits the pixels in the image into various categories one at a time based on one or more thresholds, and the value of the threshold is decided based on the gray level [8, 10]. The fundamental objective of image binarization is to segment those regions of the image that have areas of the same gray level. This is done so that each area of the same gray level can be assigned to a distinct category in the source image. All of the pixels in one particular gray-level region share the same attribute qualities, but the pixels in other gray-range regions do not have this property [12].

Only the grayscale information contained inside the image is utilized in the threshold-based segmentation method, which results in the algorithm having a relatively low sensitivity to background noise. Because of this, the segmentation result produced by the threshold segmentation approach will be quite unsatisfactory whenever the gray values of the regions that are to be segregated are comparable to one another. There are many different types of brain tissues visible in medical pictures of the human brain. Because of the complicated nature of the characteristic intensity distribution in the photos, it will be quite challenging to choose a suitable threshold value. If you solely utilize the threshold segmentation approach, it will be tough to obtain the desired impact of segmentation because of the intricacy. As a result of this, academics frequently mix threshold-based algorithms with other methods in order to successfully accomplish the task of medical image segmentation. In their study [14], Sandeep and colleagues suggested a sparse feature threshold that was based on compressed sensing, and they utilized it to segment gray matter and white matter in MRI images of the brain. It begins by training a sparse dictionary that is appropriate for the corresponding image, then employs compressed sensing technology to extract the sparse features of the image patch that correspond to the pixel point, and finally applies the sparse projection threshold to the image in order to segment it and obtain a variety of binary images.

The edge-detection-based segmentation approach first extracts the pixels that mark the boundaries of the various image sections and then links each of the collected pixels individually. The segmented region has a boundary that is represented by the connection line. The performance of this approach is satisfactory for evident areas that have a straightforward background. However, when confronted with images that are rich in features and have uneven brightness, such as MRI scans of the human brain, the edge detection approach finds it challenging to entirely detect the edge pixels of the object area. As a result, it is unable to accomplish reliable object segmentation. When doing region segmentation, particularly when employing hard-means to separate pixels, this will almost always result in the image being oversegmented [16]. Some researchers have suggested using fuzzy clustering methods as a solution to these kinds of issues. The fuzziness of classification is described by fuzzy c-means clustering through the application of membership function, which may more accurately and scientifically characterize the pixels in the image that are located in the intersection area of two different categories. The fuzzy c-means clustering method is extremely sensitive to noise; hence, it is particularly well suited for the segmentation of images with low levels of noise. Additionally, the training speed may be very slow when it is employed in clustering situations that include a big quantity of data; the selection of the initial center point has a significant impact on the amount of work that is required. The quantity of calculations will dramatically increase when there is a little bigger variation between the initial center point and the ground-truth center point. In addition, with this method of clustering, it is impossible to avoid falling into a situation where a local optimum has been reached. Kandan and Murugeswari [18] devised a novel approach to complete the segmentation of medical MRL brain pictures. This algorithm is based on the FCM algorithm, which was designed to improve the aforementioned difficulties. The genetic algorithm and the particle swarm optimization method are utilized in order to locate the initial center point that is optimal for the situation. In addition, the FCM algorithm is particularly vulnerable to noise due to the fact that it only analyzes the gray value between pixels. However, the new approach reconstructs and optimizes the objective function, which makes it acceptable for noisy MRI brain pictures. The fundamental concept behind the level-set approach is to employ the development of three-dimensional surfaces to symbolize the development process of two-dimensional curves. This is done by using a level set. In the realm of computer vision, the level set approach has the potential to produce satisfactory results when applied to picture segmentation. An improved spatial fuzzy clustering level set segmentation algorithm was proposed by Yuan and Yu [19] for MRI brain tissue segmentation. The Neumann boundary condition of the third function of level set evolution is combined with this method, and then, that boundary condition is used to obtain the directional derivative of the normal of the specified function on any surface.

The fundamental concept behind the level set technique is to model the development of two-dimensional curves by simulating the growth of three-dimensional surfaces [20]. The level-set method, which is used in the field of computer vision, is capable of producing high-quality results when segmenting images. An enhanced version of the spatial fuzzy-clustering level-set technique was proposed by Parker and Feng [21] for the purpose of MRI brain tissue segmentation. To calculate the directional derivative of the normal of the supplied function on any surface, this method combines the Neumann boundary condition with the third function of level-set evolution. Start from a specific pixel or a small region as the starting point for the region-growth method. Merge the pixels or regions near it that have characteristics that are similar to the growth point in order to form a new growth point. Then, repeat the growth process until the growth conditions are no longer satisfied. An algorithm that segments MRI brain tissue in phases and is based on the expansion of regions was proposed by Kuo et al. [22]. However, the segmentation effect of scattered cerebrospinal fluid is not very good.

In recent years, academics from all around the world have come up with a variety of segmentation algorithms. Because of this, the MRI brain tissue segmentation program allows for the selection of a large number of different segmentation techniques. Every approach has perks and drawbacks of its own, and the circumstances in which they are most useful are rarely the same [23, 24]. According to the preceding analysis, the clustering-based segmentation algorithm achieves better results when applied to the process of brain tissue segmentation. However, the clustering-based algorithms also include K-means clustering, fuzzy c-means clustering, maximum entropy clustering, Gaussian mixture model, mean-shift, and agglomerative cluster. The effectiveness of each of these algorithms for clustering data likewise varies to varying degrees. In order to determine which clustering algorithm is the most effective for MRI brain tissue segmentation, this article will first examine a number of different clustering algorithms and then compare the performance and impacts of these various methods. The segmentation algorithm that is suited for medical brain imaging is the primary emphasis of this research. The clustering approach is also discussed briefly.

The remaining parts of the paper are structured as described below. In Section 2, we will discuss the works that are linked. The typical algorithms for grouping textures are discussed in Section 3, including the mean-shift algorithm and the fuzzy c-means algorithm. In Section 4, we conduct an analysis of the simulation model as well as the outcomes of the comparison. In the end, we bring our work to a close and then move on to Section 5, where we address future work.

## 2. Related Works

### 2.1. Difficulty of MRI Brain Tissue Segmentation

Imaging of the human brain makes extensive use of magnetic resonance imaging (MRI), which, as we all know, offers several benefits, including strong contrast in soft tissues, the absence of radiation damage, and widespread use. The segmentation of brain tissue by MRI not only contributes to the study of the function and anatomical structure of the brain, but it also offers a theoretical foundation for the diagnosis and treatment of brain illnesses [25]. Because of this, the achievement of correct tissue segmentation with MRI has a very significant impact on clinical diagnosis and therapy. Gray matter (GM), white matter (WM), cerebrospinal fluid (CSF), muscle, bones, and other important brain structures can be seen in clinical MRI brain images, as depicted in Figure 1. However, due to the fact that the human brain is highly complicated in its structure and that there are many different types of brain tissues, the human brain structure of each individual has its own set of distinctive qualities. Because of these several circumstances, the process of segmenting brain tissue will be challenging. As a result, the development of an outstanding segmentation algorithm that is appropriate for every MRI brain tissue is a topic that presents a significant amount of difficulty. While doing so, it also encourages the research of brain tissue segmentation algorithms and has become a center of attention for research at the present time. In clinical practice, it is frequently required to present a three-dimensional model of the structure of brain tissue in order to offer a foundation for the diagnosis and treatment of a patient. For instance, if brain surgery is required, the procedure can be planned and simulated in accordance with the three-dimensional anatomy of the brain. This makes it easy for the focus to rapidly and properly determine the place of the surgery [26–28]. In addition, the goal of visualizing brain tissue is to finish the job of segmenting it, which is the concept of visualization. As a result, the process of segmenting brain tissue has significant use in the field of medical diagnosis.

The human brain is made up of several different tissues, each of which has a unique structure, as well as a different form and dimension. In the human brain, the boundary shape of white matter, gray matter, and CSF is complicated and alternatively distributed; also, the topological organization is complex [27]. Additionally, the distinctions between tissues in MRI images of the human brain are particularly visible in the disparities of gray information. In general, the gray information that is shared between various tissues has significant variances, whereas the gray information that is shared between the same tissues is identical [28]. However, in greater detail, due to the inherent signal changes in the imaging process, the same tissue will also display variances in the gray information. This results in the overlapping of the gray information of various tissues, which makes tissue segmentation more challenging. In Figure 2, the area shown in red and blue has been enlarged. It is clear that areas that fall under the same category have a complicated distribution of gray, and that some patches share the same gray scale and characteristics. When a straightforward threshold method is applied, it is challenging to partition the comprehensive tissue data.

In magnetic resonance scans of the brain, a variety of tissues can be seen, including fat, skull, and muscle. The gray information of these tissues is highly similar to the gray information of the gray matter, white matter, and cerebrospinal fluid (CSF) in the brain, which makes it more difficult to precisely segment the different types of tissue in the brain. Therefore, prior to segmenting brain tissue, it is required to exclude the tissues that do not belong to the brain in order to assure the correctness of the segmentation. This is done so that the segmentation will be accurate. The elimination of nonbrain tissue, on the other hand, is a challenging procedure, which makes the segmentation of brain tissue much more difficult. The uniformity of each tissue and the continuity of the boundary are destroyed, which leads to an unsatisfactory segmentation effect and a reduction in segmentation accuracy. Additionally, the distribution of gray information changes as a result of the influence of electrical noise, which appears as salt-and-pepper noise or Gaussian noise. Based on the study shown above, it is clear that successfully segmenting human brain MRI images is a challenging task. As a result, the question of how to accurately segment human brain MR images remains a contentious and challenging one in the field of medical image processing.

### 2.2. Clustering Analysis

Within the realm of artificial intelligence, the clustering algorithm is an essential component of the unsupervised learning methodology. It is an efficient method for analyzing data, extracting useful information from data, and classifying data. In addition, clustering analysis technology can divide individuals with similarity into the same cluster/subset by calculating the similarity between samples in the dataset. This is accomplished by calculating the correlation between the samples in the dataset. In this context, each subset is referred to as a cluster, and inside each cluster, there is exactly one cluster center.

Clustering algorithms can be loosely broken down into two distinct categories: those that work at the pixel level and those that work at the feature level. The first category includes hierarchical clustering, partitioned clustering (K-means and FCM), and density-based partitioning (GMM); feature-level clustering has become a popular research direction in recent years; the second category includes constraint-based partitioning, fuzzy-based partitioning, granularity-based partitioning (mean-shift), kernel clustering, and spectrum clustering; all of these are illustrated in Figure 3. In recent years, the majority of the algorithms that are used for the segmentation of brain tissue are based on K-means clustering, fuzzy c-means clustering, maximum entropy clustering, Gaussian mixture model, mean-shift, and hierarchical cluster. K-means clustering is an acronym for “Kernel means clustering.” Rarely are corresponding investigations carried out on the performance of all clustering methods on the same data set in order to determine the adaptability of the algorithms. In the following part, we will go over the typical algorithms in further detail.

## 3. Typical Clustering Algorithm

Recently, scholars at home and abroad have proposed many clustering-based segmentation algorithms. Therefore, a wide variety of segmentation techniques can be selected in the application of MRI brain tissue segmentation. Each clustering algorithm has its advantages and disadvantages, and the practical situations are also different, where mean-shift and fuzzy c-means clustering are representative algorithms. We will introduce these two algorithms for clustering in detail.

### 3.1. Fuzzy c-Means Clustering

The fuzzy c-means algorithm (FCM) is the most widely used clustering approach in the field of picture segmentation. The FCM algorithm is a method for the clustering of data that is based on the optimization of an objective function. A numerical value is used to indicate the degree of membership that each sample has in the clustering center. It is permissible for a sample to have the same numerical value and still belong to numerous distinct classes. The FCM algorithm is a method of unsupervised clustering that does not take into account the influence of human factors. As a result, the investigation into the division of brain tissues is extremely significant. It uses an iterative method to constantly update the cluster center and constantly optimize the objective function, which causes the objective function to reach the least value and classifies the pixels using the maximum membership criterion. This is the fundamental concept behind it. The following is a textual representation of the objective function of the FCM algorithm:

(1) $$\begin{array}{c} J=\overset{c}{\underset{k=1}{\sum }}\overset{N}{\underset{j=1}{\sum }}\mu_{kj}^{m}{\left\|x_{j}-v_{k}\right\|}_{2}^{2}, \end{array}$$

where *N* is the number of pixels in the image; *x*_*j*_ is the *j*-th pixel point; *c* is the preset number of clusters; *v*_*k*_ is the *k*-th cluster center; *m* is the fuzz factor; *u*_*kj*_ is the membership degree of the *j*-th sample point the *k*-th cluster. For any pixel *j* and its class *k*, there are the following constraints:

(2) $$\begin{array}{c} \overset{c}{\underset{k=1}{\sum }}u_{kj}=1,0\leq u_{kj}\leq 1. \end{array}$$

Generally speaking, the Lagrange multiplier method is used to solve the above formula (Equation (1)) with constraints, and the formulas for updating the membership degree and cluster center are given as follows:

(3) $$\begin{array}{c} \mu_{kj}=\frac{1}{\sum_{k=1}^{c}{\left({\left\|x_{j}-v_{k}\right\|}^{2}/\left\|x_{j}-v_{l}\right\|\right)}^{1/m-1}}, \end{array}$$

(4) $$\begin{array}{c} v_{k}=\frac{\sum_{j=1}^{N}\mu_{kj}^{m}x_{j}}{\sum_{j=1}^{N}\mu_{kj}^{m}}, \end{array}$$

where *u*_*kj*_ is the membership degree of the *j*-th sample point the *k*-th cluster and *v*_*k*_ is the cluster center. Through the above two equations, the membership of the cluster center *v* and the pixel point *x* is repeatedly updated, and finally, the segmentation result can be completed and achieved when the objective function reaches the convergence criterion. Generally, whether the objective function reaches the minimum value can be judged by the difference between the objective functions in the two iterations being less than the error threshold value, but it is easy to fall into the local optimal solution. Therefore, the fuzzy c-means algorithm usually takes the maximum change value of the pixel membership or the maximum change value of the cluster center as the condition of the end of the iteration.

The algorithm steps are given as follows:

1. Set the number of cluster centers *c*
2. Randomly initialize the cluster center *v*_*i*_
3. Use the corrected cluster center matrix to update the membership matrix
4. Utilize the corrected membership degree matrix to update the cluster center matrix

The preceding analysis demonstrates that, similar to the K-means algorithm, the number of cluster centers for the FCM algorithm needs to be given in advance; however, the number of clusters in an MRI image is typically unknown in practical applications. This can be seen from the fact that the above analysis was performed. The clustering effect will be greatly reduced when the initial value or preset value is not equal to the ground-truth value. Secondly, according to Equations (3) and (4), it can be seen that the FCM algorithm is an iterative operation on basis of gradient descent, so it is also very sensitive to the initial value. This is because the FCM algorithm is based on the principle of gradient descent. In addition, random initialization makes it quite simple to get stuck in a cycle of local optimization, which in turn results in a reduction in the estimation accuracy of the final segmentation results.

The FCM algorithm is more reliable than the K-means algorithm because it includes a fuzziness factor when describing each data sample. K-means does not include this component. The accuracy of the FCM algorithm will be higher than that of the K-means algorithm when applied to the brain tissue clustering; however, due to the introduction of membership factor, the objective function is more complex, so the complexity of the FCM algorithm is higher than that of the K-means algorithm. For the clustering of each sample, it will be more accurate than the traditional K-means hard clustering. When applied to the brain tissue clustering, the segmentation speed can be slower than that of the K-means algorithm.

### 3.2. Mean-Shift Clustering

Mean-shift is a kind of density clustering algorithms, which belongs to a specific theory for image segmentation when used as a segmentation method. Since mean-shift uses the density gradient method to estimate the parameters of distribution and uses the kernel function to weight the samples in mean-shift clustering. When allocating weights to the samples in each bandwidth, the contribution of the offset to the mean-shift vector varies with the distance between the samples and the offset. Mean-shift assumes that the datasets of different clusters conform to or obey other probability density distributions. By finding the densest direction in the sample set and constantly shifting to the maximum density, it is considered that the point converging to the same maximum in the iterative process is a member of the same cluster as the sample converges to the local density maximum.

Given *n* sample points in *dd*-dimensional space *R*^*d*^, the mean-shift vector at the point *x*_*i*_ can be denoted as

(5) $$\begin{array}{c} M_{h}\left(x\right)=\frac{1}{k}\underset{x_{i}\in S_{h}}{\sum }\left(x_{i}-x\right), \end{array}$$

where *M*_*h*_(*x*) is the mean-shift vector, *S*_*h*_ is a high-dimensional sphere with a radius *h*, *x*_*i*_ represents the sample points in the high-dimensional sphere region, and *x* represents the initial clustering center point; *k*means that *k* points fall into the region *S*_*h*_ among the *n* sample points; Equation (5) is to calculate the average value of the sample weight in the high-dimensional ball, where *x*_*i*_ close to point *x* should have a higher weight. Introducing the kernel function and *ω*(*x*_*i*_) to weight the samples in mean-shift, the mean-shift clustering is extended to the following form:

(6) $$\begin{array}{c} M_{h}\left(x\right)=\frac{\sum_{i=1}^{n}G\left(\left(x_{i}-x\right)/h\right)\omega \left(x_{i}\right)\left(x_{i}-x\right)}{\sum_{i=1}^{n}G\left(\left(x_{i}-x\right)/h\right)\omega \left(x_{i}\right)}, \end{array}$$

where *ω*(*x*_*i*_) > 0 is a weight assigned to sample point *x*, *G*(*x*) is the unit kernel function, and *G*(*x*) = ‖*x*‖^2^ is the bandwidth of the kernel function. Gaussian kernel function is often used in brain tissue segmentation.

If the weight *ω*(*x*_*i*_) is not considered in Equation (6), the mean-shift vector between the cluster center and the sample *x*_*i*_ in the bandwidth can be rewritten as follows:

(7) $$\begin{array}{c} M_{h}\left(x\right)=\frac{\sum_{i=1}^{n}G\left(\left(x_{i}-x\right)/h\right)x_{i}}{\sum_{i=1}^{n}G\left(\left(x_{i}-x\right)/h\right)‐x}. \end{array}$$

Let *m*_*h*_(*x*) = ∑_*i*=1_^*n*^*G*((*x*_*i*_ − *x*)/*h*)*x*_*i*_/∑_*i*=1_^*n*^*G*((*x*_*i*_ − *x*)/*h*), and Equation (4) can be rewritten as follows:

(8) $$\begin{array}{c} m_{h}\left(x\right)=M_{h}\left(x\right)+x \end{array}$$

*m*_*h*_(*x*) is the new cluster center after *x* plus *M*_*h*_(*x*). In MRI brain tissue segmentation, the gray values of the same cluster are selected, and then, the regions less than *M* pixels are merged. The final segmentation result is obtained through iterative optimization. The essence of mean-shift is to solve the local maximum of probability density, where the mean-shift vector makes the object point always move to the maximum point of probability density. Therefore, a region near the object point is often selected for greedy iteration, gradually converging the maximum probability density.

## 4. Experiment Results and Analysis

This paper selects ten brain images from a simulated brain database, which contains a set of realistic MRI data volumes produced by an MRI simulator and can be downloaded from https://brainweb.bic.mni.mcgill.ca/. The purpose of this selection is to make it easier to compare the results of different experiments. To begin, six standard clustering techniques are picked to segment MRI brain pictures. Next, two evaluation indexes are chosen to compare the performance of these comparison algorithms. Finally, the results of this comparison are presented. In the final step, the qualitative and quantitative outcomes produced by the various algorithms are compared and examined.

### 4.1. Comparison Algorithm Selection

In recent years, academics from all around the world have come up with a variety of segmentation algorithms. Methods that are partition-based, density-based, grid-based, and constraint-based are the broad categories that can be used to classify the clustering algorithms. The clustering algorithm is being used more frequently, and as a result, it is putting forward stronger requirements for itself. This is because research is becoming more in-depth, and the morphology of data is becoming more diverse. In order to cluster brain tissue, these algorithms make use of a variety of different clustering principles and procedures; yet, the results that they produce are satisfactory.

As a consequence of this, the application of MRI brain tissue segmentation allows for the selection of a wide variety of different segmentation approaches. Each approach has a unique set of benefits and drawbacks, and the circumstances in which they are most useful are never the same. However, clustering-based segmentation algorithms encompass a wide variety of subcategories, despite the fact that their performance is superior in brain tissue segmentation. The effectiveness of each of these techniques for clustering likewise varies to varying degrees. As a result, we chose six different clustering techniques to compare and contrast: the K-means clustering algorithm, the fuzzy c-means algorithm, the Gaussian mixture model, the mean-shift algorithm, the fuzzy subspace clustering strategy, and the maximum entropy clustering algorithm. To determine which MRI brain tissue segmentation method is superior in the long run, each algorithm's effectiveness in clustering brain tissue and its effect on segmentation are evaluated independently.

### 4.2. Parameter Setting and Development Platform

In the field of medical image processing, image segmentation is the process of dividing a picture into many mutually distinct sections based on the anatomy structure. This approach makes use of the fundamental characteristics of the image, such as gray scale and texture. In a perfect world, the outcomes of the segmentation would be such that each region would be able to take into account both the similarity of pixels between regions as well as the homogeneity of pixels within its own region. The segmentation of brain tissue MRIs is the primary focus of this particular piece of research. There are four distinct types of brain tissue, which are referred to as white matter, gray matter, cerebrospinal fluid, and other tissues. For this reason, the number of clusters in all comparison algorithms is always set to 4.

On the other hand, the initial clustering center of the clustering algorithm is generated in a random manner, and these initial values may contain nondense points or abnormal points. This results in the clustering algorithm falling into the local extremum, which in turn lowers the segmentation accuracy. In addition, the initial value may be rather removed from the actual center of clustering, which results in an increase in the number of iterations required for clustering and a decrease in the algorithm's effectiveness. In order to make comparative analysis easier, this study uses the source code to evaluate the six traditional comparison techniques that were chosen for inclusion in it. Additionally, all of the parameters are set to their default settings, and the initial values are determined using random number seeds. Normalized Mutual Information (NMI) and Rand Index (RI) are adopted to analyze the performance of comparison algorithm, where all quantitative results are the average of five experiments in order to reasonably and fairly evaluate the clustering performance of each clustering algorithm. This is done in order to reasonably and fairly evaluate the clustering performance of each clustering algorithm. These two indicators have a value range of [0, 1], and the general rule of thumb is that a greater number indicates a higher level of clustering performance.

These cluster methods are implemented in MATLAB on Windows 10 with a 64-bit system, and the hardware platform is on a Windows PC equipped with Intel(R) Core(TM)i5-1135G7 CPU@2.50 GH and 4 G RAM.

### 4.3. Qualitative Analysis of Different Algorithms

Ten brain MRI samples are chosen at random from the BrainWeb database in order to test the full segmentation performance of various clustering techniques. Because of the confines of the available area, we will only be analyzing a select few examples of typical image segmentation findings. For the MRI brain tissue to preserve its precise information, the clustering technique is required. This is due to the complicated structure of the tissue. Therefore, in order to conduct a comparative analysis of various algorithms, the research applies the clustering algorithms that were selected to the segmentation of MRI brain tissue. The results of the segmentation performed by the various algorithms are displayed in Figures 4 and 5.

In human brain magnetic resonance scans, there are many structural tissues that do not belong to the brain, such as fat, the skull, muscle, and other tissues. Because the gray information of these tissues and the gray information of particular brain structures are so highly comparable to one another, proper segmentation of brain tissues is made more difficult as a result. Therefore, when segmenting brain tissue, it is required to exclude the tissues that do not belong to the brain in order to assure the correctness of the segmentation. This is done to ensure the correctness of the segmentation. Nevertheless, the procedure of removing tissue that is not part of the brain is challenging and complicated. In this study, the nonbrain tissues have been grouped together under the same category or cluster. Figures 4 and 5 show the segmentation results, which show that the segmentation results of the K-means clustering algorithm have a lot of noise, the segmentation results of the FCM algorithm contain a small amount of noise in white matter and cerebrospinal fluid, and the segmentation results of the hierarchical cluster algorithm remove the noise, but the cerebrospinal fluid in the brain sulcus is also smoothed out. These results can be seen by looking at the segmentation. On the other hand, the results of the mean-shift algorithm's segmentation are the most accurate of all of them. Despite the fact that Figures 4 and 5 demonstrate the results of segmentation using different methods, they are unable to portray the results of distinct tissues in a way that is intuitive. As a result, the experiment provides evidence of the segmentation outcomes of several categories. The benchmark of several different types of tissues in the selected image is shown in the first row of Figures 6–11. The remaining rows of the figure contain the clustering results corresponding to K-means clustering, fuzzy c-means clustering, maximum entropy clustering, Gaussian mixture model, mean-shift, and hierarchical cluster, making it easy to compare the clustering results produced by various algorithms. The K-means clustering technique is discovered to have flaws when they are compared to other algorithms, and the results of the clustering are found to be largely one-sided, meaning that they can only segment a portion of the region.

A comprehensive white-matter region cannot be obtained using maximum entropy clustering. Both the hierarchical cluster method and the Gaussian mixture model algorithm are capable of obtaining a white-matter region that is relatively comprehensive; however, the boundary part of the gray-matter region does not appear to be particularly obvious. When compared to previous techniques, the white-matter region generated by the fuzzy c-means clustering approach is both more complete and more transparent.

It has been demonstrated through observation that it is challenging for each comparison method to achieve a decent segmentation effect for MRI brain pictures that contain four clusters. The white-matter region of some clustering methods has a significant number of incorrectly categorized pixels, which not only has a negative impact on the region's overall integrity but also produces an unsatisfactory aesthetic effect. The FCM algorithm increases the impact of the cerebrospinal fluid (CSF) when compared to the K-means algorithm; nonetheless, there are still some scattered misclassifications, and the outcome needs further development. Visually, the FCM method achieves the best segmentation effect; nevertheless, for some photos, the mean-shift approach achieves the best results. All of the results from the MRI segmentation have the consistency of homogeneous regions, and they do a better job of preserving the border information. There are no obviously incorrect pixels in any of these findings.

It is clear from the results of the segmentation that FCM has high robustness and obtains more accurate segmentation results. While the K-means algorithm is able to segment white matter, the results of segmenting gray-matter regions are substantially worse. In contrast, the FCM is significantly larger than the other approaches, and it produces more accurate segmentation results. When compared to the other cluster algorithms shown in Figures 6–11, the FCM has the highest segmentation performance thanks to its superior accuracy when it comes to the segmentation of various MRI brain pictures. When calculating the pixel similarity, all traditional clustering algorithms only take into account the gray information of the image. This results in severe interference from noise and uneven gray in the process of segmentation, which is something that should be brought to your attention. The precision of the segmentation is not very great, and the details of the edge of the tissue that has been segmented are not very visible. On the other hand, it is necessary for each algorithm for clustering to do an initialization of the clustering center beforehand. The initial clustering center, for instance, is generated in a haphazard manner by the traditional FCM algorithm. When the initialization is poor, it is difficult for the algorithm to converge rapidly, it takes a long time to run, and it even leads to the algorithm easily falling into the local optimal point, which impacts the clustering accuracy. All of these problems arise because of the poor initialization. It is important to note that the equivalent class in Figures 6(c), 7(e), 8(e), 9(e), 10(b), and 11(d) does not have any detailed information. This suggests that the clustering technique does not segment the item in these classes. As an illustration, the K-means algorithm does not divide the area denoted by “gray matter” in Figure 6.

As can be seen from Figures 6–11, since the FCM algorithm only uses grayscale information to calculate the similarity between pixels, there are still many misclassification points in the segmentation result, and the tissue boundary is not clear. The optimal initial clustering center of the maximum entropy clustering algorithm reduces the noise points compared with the FCM algorithm, but the segmentation result is still poor. Although the image segmented by the Gaussian mixture model algorithm has fewer noise points, the edge details of each tissue are incomplete. For example, when segmenting gray matter, the background details are wrongly segmented, and the segmentation effect is not good. The tissue images obtained by these algorithms are different from the benchmark images. The edge details are not very complete, and the segmentation effect is not perfect. However, it is undeniable that these traditional clustering algorithms do not require pretraining, have little computation, and are easy to deploy in the brain tissue application.

### 4.4. Quantitative Analysis of Different Algorithms

From the segmentation result, it can be seen that the FCM algorithm has less noise points in the segmented image, and the edges of the segmentation image are clearer. The performance of the algorithm is better, and the reliability is higher.  Table 1 shows the quantitative results of different algorithms. It can be seen that the FCM algorithm has higher segmentation accuracy than the comparison algorithm.

The FCM algorithm for the segmentation of cerebrospinal fluid has relatively high NMI and RI indexes, but the average index is quite low. RI-mean of FCM is 0.89931, while that of mean-shift is 0.90666. To put it another way, the RI-mean of the FCM is not the ideal option because the mean-shift algorithm has a high segmentation index for the white matter of some images. It can be seen from the assessment indicators in Table 1 that FCM is optimized in terms of segmentation accuracy compared with the prior algorithms, and the final average segmentation accuracy is 0.73121 and 0.89931, respectively. Compared with the K-means, MEC, GMM, HC, and mean-shift algorithms, the NMI index of FCM algorithm is increased by 1.86 percent, 2.07 percent, 1.83 percent, 1.13 percent, and 0 69 percent, and RI index rose by 1.66 percent, 1.69 percent, 1.44 percent, 0.46 percent, and 1.26 percent. On some images, the mean-shift algorithm produces the best results, while the FCM clustering algorithm produces the best results on other images. Mean-shift does not need to manually set the number of clusters; hence, the segmentation effect on some photos is significantly better than other techniques.

In general, the FCM method is better than these comparison algorithms, which enhances the performance of K-means algorithm on the whole. FCM algorithm has better consistent performance and higher universality. It can better segment brain images and effectively resist some interference, which has higher performance when segmenting images with complex backdrops.

## 5. Conclusions

As a result of the high level of complexity that the human brain possesses as well as the wide variety of different types of brain tissues, the physical composition of the human brain differs from person to person. Because of these several circumstances, the process of segmenting brain tissue will be challenging. In this article, several different clustering algorithms will be discussed, and their performance and effects will be compared to one another. The goal of this comparison is to determine which algorithm is most suited for segmenting MRI brain tissue. The segmentation algorithm that is suited for medical brain imaging is the primary emphasis of this research. The clustering approach is also discussed briefly. The qualitative and quantitative findings of the experiment reveal that the FCM algorithm has more steady performance and higher universality, but the addition of the auxiliary conditions is necessary in order to produce outcomes that are closer to being perfect.

In the future, we are going to conduct additional research into the efficacy of deep learning networks in the segmentation of brain tissue, compare and contrast it with the performance of traditional algorithms, and investigate the degree to which traditional algorithms and intelligent algorithms are adaptable.

## Figures and Tables

**Figure 1:** Tissue segmentation of human brain. (a) Raw image; (b) segmentation result; (c) white matter; (d) gray matter; (e) CSF.

**Figure 2:** Grayscale difference among different tissues.

**Figure 3:** Classification diagram of clustering algorithm.

**Figure 4:** Comparison of clustering results of different algorithms for Figure 1.

**Figure 5:** Comparison of clustering results of different algorithms for Figure 8.

**Figure 6:** Clustering results of K-means algorithm for different tissues. (a) Clustering results; (b) CSF; (c) GM; (d) WM; (e) other tissue.

**Figure 7:** Clustering results of FCM algorithm for different tissues. (a) Clustering results; (b) CSF; (c) GM; (d) WM; (e) other tissue.

**Figure 8:** Clustering results of MEC algorithm for different tissues. (a) Clustering results; (b) CSF; (c) GM; (d) WM; (e) other tissue.

**Figure 9:** Clustering results of GMM algorithm for different tissues. (a) Clustering results; (b) CSF; (c) GM; (d) WM; (e) other tissue.

**Figure 10:** Clustering results of mean-shift algorithm for different tissues. (a) Clustering results; (b) CSF; (c) GM; (d) WM; (e) other tissue.

**Figure 11:** Clustering results of HC algorithm for different tissues. (a) Clustering results; (b) CSF; (c) GM; (d) WM; (e) other tissue.

**Table 1:** Quantitative results of different algorithms.

Images	Indexes	Clustering models					
		K-means	FCM	MEC	GMM	HC	Mean-shift
1	RI	0.8899	0.8914	0.8898	0.8855	0.8569	0.8976
	NMI	0.7131	0.715	0.7135	0.7059	0.6421	0.7289
2	RI	0.8889	0.8911	0.8878	0.8851	0.8834	0.8947
	NMI	0.7107	0.7147	0.7091	0.7049	0.6944	0.691
3	RI	0.8915	0.894	0.8915	0.8873	0.878	0.9023
	NMI	0.7163	0.7202	0.7162	0.7099	0.6993	0.7108
4	RI	0.896	0.898	0.896	0.8917	0.8783	0.9062
	NMI	0.7262	0.7292	0.7262	0.7188	0.6792	0.7228
5	RI	0.8983	0.9007	0.8984	0.896	0.9003	0.9143
	NMI	0.731	0.7355	0.731	0.7283	0.7133	0.7373
6	RI	0.9012	0.9026	0.9012	0.8971	0.896	0.9039
	NMI	0.7371	0.7399	0.7371	0.7307	0.7184	0.7412
7	RI	0.9005	0.9017	0.9005	0.8951	0.8992	0.9071
	NMI	0.732	0.7339	0.732	0.7238	0.7062	0.7446
8	RI	0.902	0.9031	0.902	0.895	0.8923	0.9148
	NMI	0.7362	0.7375	0.7362	0.7234	0.7125	0.7061
9	RI	0.9028	0.9052	0.9028	0.8964	0.901	0.9137
	NMI	0.7391	0.7423	0.7391	0.7291	0.7342	0.7369
10	RI	0.9039	0.9053	0.9039	0.8959	0.8931	0.912
	NMI	0.7418	0.7439	0.7418	0.7288	0.7245	0.7569
Average	RI-mean	0.8975	0.89931	0.89739	0.89251	0.88785	0.90666
	RI-std	0.005316	0.005131	0.005516	0.004524	0.0131775	0.00674436
	NMI-mean	0.72835	0.73121	0.72822	0.72036	0.70241	0.72765
	NMI-std	0.010719	0.010418	0.010946	0.009479	0.024977688	0.01903099

## Data Availability

The dataset used to support the findings of this study are available from the corresponding author upon request.
